RETRACTED

# Meta-Analysis of the Effectiveness and Safety of Glucocorticoid for the Treatment of IgA Kidney Disease

**DOI:** 10.1155/2022/5466331

**Published:** 2022-03-07

**Authors:** Jieqiong Sun

**Affiliations:** Nephrology Department, First People's Hospital of Linping District, Hangzhou, China

## Abstract

**Purpose:**

To explore the effect of glucocorticoid on immune globulin A (IgA) nephropathy by meta-analysis.

**Method:**

Search the data and literature libraries of ScienceDirect, EBSCO, Wiley, PubMed, CBMdisc, and CNKI and collect the literature on the treatment of IgA nephropathy with glucocorticoids as randomized controlled trials published at home and abroad from 1995 to 2021. The standardized mean difference (SMD) and 95% confidence interval (*CI*) were calculated by fixed-effects model. RevMan 5.0 software was used for meta-analysis of the subgroups of overall curative effect, different degree of proteinuria, different course of treatment, different creatinine level, and combined ACEI.

**Result:**

① The overall efficacy of glucocorticoid in the treatment of IgA nephropathy was better than that in the control group (*P* = 0.00001). ② The efficacy of glucocorticoid treatment in patients with IgA nephropathy with proteinuria greater than 1.50 g/d and less than 1.50 g/d was better than that in the control group (*P* < 0.01). ③ For IgA nephropathy patients with serum creatinine less than 1.50 mg/dl, the curative effect of glucocorticoid treatment was better than that of the control group (*P* < 0.01). ④ The effects of short-term treatment (<1 year) and long-term treatment (≥1 year) with glucocorticoid were better than those in the control group (*P* < 0.01). ⑤ The effect of hormone combined with ACEI drugs on IgA nephropathy was more significant (*P* < 0.01).

**Conclusion:**

The overall efficacy of glucocorticoid in the treatment of IgA nephropathy is accurate. Hormone treatment is effective for different degrees of IgA nephropathy. Considering that there is no significant effect on the efficacy of different courses of treatment, it is suggested that the course of hormone treatment can be appropriately shortened. Hormone combined with angiotensin-converting enzyme inhibitors (ACEI) can reduce proteinuria more effectively than ACEI drugs alone.

## 1. Introduction

IgA nephropathy (IgAN) is a glomerulonephritis characterized by the diffuse deposition of IgA or IgA based immunoglobulin in the glomerular mesangial area. It is a primary glomerular disease proposed by Berger and Hinglais in 1968. Today, it is the most common, accounting for more than 40.00% of primary glomerular diseases. It is the main cause of end-stage renal disease (ESRD). There are many inducements such as upper respiratory tract infection before the onset of the disease. The clinical manifestations are diverse, the duration of the disease varies, and the pathogenesis is not completely clear. At present, there is still a lack of effective treatment methods. IgA nephropathy is more and more common in young people, with a male to female ratio about 2 : 1. It has become one of the common causes of ESRD (end-stage renal failure) in young people. Worldwide, the annual incidence rate is increasing. Every 10 years, about 20.00%–30.00% of patients suffer from renal failure, and every 40 years will reach more than 40.00%.

RETRACTED

There are significant differences in clinical manifestations, pathological changes, and prognosis of IgA nephropathy. If the disease cannot be controlled in time, it may aggravate the risk of progression of nephropathy. At present, there is no specific treatment. The overall treatment goal is to reduce proteinuria, control blood pressure, slow down the progress of kidney disease, and delay the occurrence of ESRD. At present, it is considered that massive proteinuria, hypertension, continuous hematuria, obvious impairment of renal function, hyperuricemia, and renal pathological changes are clinical indicators of poor prognosis. Glucocorticoids have anti-inflammatory, antiallergic, and immunosuppression effects and are widely used in the treatment of immune-mediated inflammatory response, including kidney disease. Glucocorticoid treatment has been widely used in clinic [1]. At present, the clinical practice guidelines of the global organization for improving the prognosis of renal diseases (KDIGO) are mostly used to guide clinical work. However, due to the diversity of treatment schemes and prognostic indicators, many disputes have been caused, such as whether glucocorticoid treatment is used for moderate proteinuria IgA renal disease and whether ACEI drugs combined with glucocorticoids can treat IgA nephropathy [2]. Proteinuria is the key factor determining the prognosis of IgA nephropathy. Clinical trials are mostly conducted with single center and small samples to evaluate the prognosis. Due to large limitations and many influencing factors, the reliability of the conclusion will be low.

Therefore, we collected and sorted out the relevant research data published at home and abroad, superimposed the sample size, used proteinuria efficacy index to evaluate the risk of progression of kidney disease from different gradients, and studied the efficacy and safety of glucocorticoid in the treatment of IgA nephropathy.

### 1.1. Different Courses of Glucocorticoids in the Treatment of IgA Nephropathy

In the process of hormone treatment of IgA nephropathy, due to the different individual differences of patients, the course of hormone treatment is different. At present, there are few clinical studies on the course of hormone treatment, and there is still no unified standard to suggest the best course of hormone treatment. As early as 1986, Lai kn et al. observed that the average use of hormone in patients with IgA nephropathy for 36 months can effectively reduce the excretion of urinary protein, but it is not beneficial to protect renal function [2]. The recent test of Katafuchi R. suggested that the use of hormone for 24 months and follow-up for 60 months can effectively reduce the excretion of urinary protein, but the other effects are not obvious [3]. In 1996, Kobayashi Y. used it for 18 months [4]. The results showed that it could reduce proteinuria and protect renal function in patients with IgA nephropathy. The study of Locatelli F. found that hormone treatment for 6 months can also effectively reduce proteinuria and protect renal function. Although there are few clinical trials on the course of hormone use, they all suggest that hormone treatment can improve proteinuria, but there is some debate on the effect of long-term hormone use on renal function. Therefore, considering many side effects of hormone use, it is suggested that clinicians should be careful in the course of hormone use. Further large sample experiments are needed for confirmation.

RETRACTED

### 1.2. Hormone Treatment of Different Degrees of Proteinuria IgA Nephropathy

At present, there is still no unified standard for the classification of proteinuria in IgA nephropathy. Most of the studies believe that the 24-hour urinary protein quantitative <1.00 g/d is mild proteinuria, and >3.00 g/d is severe proteinuria, with moderate proteinuria [5]. The 2011 guidelines for the diagnosis and treatment of IgA nephropathy of the global organization for improving the prognosis of kidney diseases (KDIGO) also described the principle of the degree of proteinuria according to the above standards. However, the use of hormones in the treatment of different degrees of proteinuria is still controversial. Uzu T., Locatelli P., and Kobayashi Y. used hormone combined with antiplatelet drugs and antihypertensive drugs for treatment of IgA nephropathy with moderate proteinuria. Hormone can effectively prevent the progression of moderate proteinuria IgA nephropathy. It can reduce the level of proteinuria and prevent the deterioration of renal function. Locatelli F. explained the side effects of hormone use. Due to insufficient sample size, short follow-up period, and lack of sufficient side effect data support, hormone treatment is still recommended in most of the cases, but large sample test and follow-up report are still needed. In 2007, Reich found a significant effect in the treatment of massive proteinuria IgA (>3.00 g/d) nephropathy. For proteinuria <1.00 g/d, the effect of hormone was worse than that in massive proteinuria IgA patients, but it does not deny that hormone application is ineffective for IgA nephropathy patients with proteinuria less than 1.00 g/d. In 1988, Kobayashi Y. gave hormone therapy to a large number of IgA patients with proteinuria (2.00–4.50 g/d). The results showed that hormone could effectively reduce proteinuria and stabilize renal function and prevent progression in patients with basically normal renal function [6].

RETRACTED

### 1.3. Hormone Combined with ACEI

In 2009, 48 patients in Manno C. trial were treated with prednisone combined with ACEI [7]. It is considered that the combination of hormone and ACEI can effectively reduce urinary protein and blood pressure and prevent the progress of IgA nephropathy. In 2009, LV JC also showed that the therapeutic effect of hormone combined with ACEI was better than that of ACEI alone [8]. Because the two studies had small samples and single-center trials, there were great differences among individual patients. Therefore, it was necessary to further carry out large-sample and multicenter validation. Reich conducted a large sample trial for hormone tracking treatment in 2007 [9]. The results showed that when proteinuria was more than 3.00 g/*d*, the decline rate of renal function indexes in patients was 25 times faster than that in patients with low-grade proteinuria (1.00 g/d). For patients with proteinuria of 0.30 g/d or between 0.30 g/d and 1.00 g/d, there is no significant difference in the changes of renal function indexes between the two after long-term application of hormone. When proteinuria is greater than 3.00 g/d, hormone treatment has achieved obvious effect, but there is no data to show that the effect of hormone treatment is not obvious in patients with albuminuria of less than 1.00 g/d. In 1994, Maschio selected patients with normal blood pressure for the test [10]. The urinary protein level of patients was maintained at 1.00–2.50 g/d and the glomerular filtration rate was greater than 90 ml/min. One side was given Fosinopril and the other was placebo. The simple application of ACEI can significantly reduce proteinuria and protect renal function [11].

### 1.4. Hormone Combined Immunosuppressant

Pozzi C. observed the treatment of hormone combined with azathioprine in patients with IgA nephropathy with urinary protein greater than 1.00 g/d [12]. The results showed that the effect of combined treatment increased the risk of adverse events (leucopenia, gastrointestinal symptoms, bacterial infection, viral infection, etc.). The effect is not as good as using hormone alone. Due to the small sample size and short follow-up period of this study, it is recommended to continue relevant trials and report long-term follow-up to determine its curative effect. Walker R. G. and Woo K. T. used cyclophosphamide, warfarin, and dipyridamole alone to treat IgA nephropathy in 1990 and 1991 [13, 14]. It was found that they had no significant effect on renal function. During 2002, Ballardie F. W. used hormone combined with cyclophosphamide in the observation group, while the control group only used glucocorticoid [15]. The results showed that the therapeutic effect of combined immunosuppressive agents is far better than that of hormone alone. Pozzi C. had an opposite conclusion [16]. Does the use of immune agents affect their effectiveness? Yoshikawan compared the efficacy of hormone + different immunosuppressive agents in 2006 [17]. One group was hormone + azathioprine, and the other group was hormone + cyclophosphamide; the analysis of comparative results is as follows: the GFR of the two groups maintained a balance, and it was difficult to distinguish the difference between the combined effects of hormones and different immunosuppressants. Therefore, whether the combined effects of immunosuppressants and hormones would be more satisfactory remains to be observed in the long-term effect.

RETRACTED

### 1.5. Combination of Hormone and Antiplatelet Drugs

The combination of hormones and antiplatelet drugs (dipyridamole and dipyridamole) in the works of Shoji T., Locatelli F., Kobayashi T., and Uzu T. can reduce urinary protein excretion [12, 18]. Due to the small sample size and short follow-up period of Shoji T.'s study, all except in Shoji T.'s work can protect renal function.

### 1.6. Others

In recent years, the meta-analysis of fish oil (03FA unsaturated fatty acid) in the treatment of IgA nephropathy has shown that fish oil can effectively reduce proteinuria but cannot prevent the progress of renal function [2]. Considering the role of fish oil and cardiovascular and cerebrovascular diseases, the application of fish oil is safe. In addition, Koike M. et al. observed that, compared with low-dose hormone treatment, anti-inflammatory treatment has not been found to effectively improve urinary protein level and protect renal function.

### 1.7. Hormone Treatment of IgA Nephropathy by Different Pathological Types

This group did not retrieve the relevant clinical randomized controlled trial literature. Most of the trial samples covered the pathological grade but mostly discussed the changes in the pathological grade after treatment, such as Shoji I., Hogg R., Koike N., and Moriyama T. in 2004. There was no significant difference in the effect of hormone treatment of IgA nephropathy on the pathological grade; it may be that there is no targeted treatment for pathological classification during the treatment, resulting in no significant change in pathological grade after treatment.

RETRACTED

KDIGO clinical practice guideline clearly points out that proteinuria is the key factor determining the prognosis of IgA nephropathy. The five meta-analyses at home and abroad and the above cases have proved that hormones can effectively reduce the level of proteinuria, but there are different conclusions on the efficacy of renal function protection. Due to the large individual differences of patients, the limited number of studies, and the early period of literature sources, the drug treatment is different from the current treatment, and there is no clinical randomized controlled trial for pathological typing treatment [19]. Thus, the standards and evidence-based evidence for hormone therapy remain imperfect. We should go further, i.e., go for a large number of randomized controlled trials and purposefully conduct multisample multicenter clinical-based trials on controversial issues to improve diagnosis and treatment.



## 2. Materials and Methods

### 2.1. Retrieval Method and Evaluation Method

ScienceDirect, EBSCO, Wiley, PubMed, CBMdisc, CNKI, and other data and literature databases were searched. Different joint searches were carried out with the keywords glucocorticoids (ster OID) and IgA/IgAN or protein (URI protein) and ACEI, and the literature was traced. The relevant literature published at home and abroad from 1995 to 2021 were collected and sorted out by means of machine inspection and manual retrieval. More than two researchers evaluated the quality of the retrieved literature according to the Cochrane Collaboration standard, including random method and blind method.

### 2.2. Inclusion Criteria

The inclusion criteria were as follows: published RCT literature at home and abroad and EGFR >50 ml/min in patients with primary IgA nephropathy confirmed by renal biopsy. The literature includes glucocorticoid treatment group. For the literature elaborated by the same author and the follow-up reports on the same subject, the most complete data and the most recent length of time shall be included. The literature observation items include proteinuria indexes and proteinuria data in standard units.

### 2.3. Exclusion Criteria

The exclusion criteria were as follows: IgA cases diagnosed by nonrenal biopsy, secondary IgA nephropathy and animal experimental data literature [20], non-RCT literature, nonstandard diagnosis and treatment, and no proteinuria index, no unified standard for proteinuria units in RCT literature, related literature published by the same author for many times, and combination with other immunosuppressants.

RETRACTED

### 2.4. Statistical Treatment

Statistical analysis was performed by RevMan 5.0 software. The final indexes were analyzed by SMD value and 95% CI. If *P* ≤ 0.01, it means that the curative effect difference is statistically significant. The test results were tested for heterogeneity and comprehensively evaluated by qualitative analysis of Q test and quantitative analysis of *I*^2^ test. If *P* > 0.10, the literature results were homogeneous, and the fixed-effects model (reciprocal weight method of variance) was used; if *P* < 0.10, there was heterogeneity, and the random-effects model (D-L method) was used; if *I*^*2*^ > 50.00% it indicated that there was heterogeneity, and descriptive systematic evaluation, subgroup stratified analysis, or metaregression was used to explore the source of heterogeneity.

## 3. Results

### 3.1. General Information and Literature Quality Analysis

#### 3.1.1. Grouping Evaluation and Index Determination

① The efficacy of glucocorticoid in the treatment of proteinuria in IgA nephropathy was evaluated. ② The efficacy of IgA nephropathy with different urinary protein was analyzed. Taking 1.50 g/d proteinuria as the baseline, the patients with urinary protein less than 1.50 g/d and patients with urinary protein greater than 1.50 g/d were evaluated, respectively. ③ The curative effect of IgA nephropathy with different blood creatinine levels was analyzed. Taking 1.50 mg/dl blood creatinine as the baseline, the patients with blood creatinine less than 1.50 mg/dl and patients with blood creatinine greater than 1.50 mg/dL were evaluated, respectively. ④ The course of treatment of IgA nephropathy with glucocorticoid was 1 year as the baseline, the short-term course of treatment with glucocorticoid was less than 1 year, and the long-term course of treatment was more than 1 year. ⑤ The therapeutic effect of combined application of ACEI on proteinuria was evaluated.

Through electronic retrieval and manual retrieval, there were a total of 935 Chinese literature, 1207 English literature, 908 cross repeated literature between databases, 27 experiments with glucocorticoid drugs as the observation group, and 19 in line with the principle of randomization, including 1 in Chinese. The literature with inconsistent index units and incomplete proteinuria data information were excluded; finally, 9 well-designed English RCTs were used for metaevaluation. 256 patients in the hormone group and 273 patients in the control group were included in the analysis, and the literature quality level was grade A.

RETRACTED

### 3.2. Overall Evaluation of the Efficacy of Proteinuria

The data of 9 literature were included, and the funnel analysis showed that 9 literature had no publication bias. The literature data were tested for heterogeneity; *P* = 0.21 > 0.10 and *I*^*2*^ = 27.00% indicated that there was homogeneity among the nine literature. The fixed-effects model was used for analysis. The results showed that the literature SMD was −0.51 and 95% *CI* was [−0.68, −0.33]; the difference was statistically significant (*P* < 0.01, see Table 1), suggesting that glucocorticoid was better than the control group in the treatment of IgA nephropathy proteinuria.

### 3.3. Efficacy Analysis of Different Degrees of Proteinuria Hormone Treatment

IgA nephropathy with proteinuria less than 1.50 g/d was analyzed. The two included literature were tested for heterogeneity: *P* = 0.24 and *I*^*2*^ = 29.00%. The literature were homogeneous. The fixed-effects model was used for analysis. The results of meta-analysis showed that the difference was statistically significant (*P* < 0.01). At the same time, there was no publication bias in funnel plot analysis. It is suggested that glucocorticoid group has obvious effect on IgA nephropathy with urinary protein less than 1.50 g/d (see Table 2). IgA nephropathy with proteinuria greater than 1.50 g/d was analyzed. The two included literature were tested for heterogeneity: *P* = 0.20 and *I*^*2*^ = 39.00%. The literature were homogeneous. The fixed-effects model was used for analysis. The results showed that the total SMD value and 95% *CI* were located on the left side of the vertical line: SMD = −0.41, 95% *CI* [−0.75, −0.07], and the difference was statistically significant (*P* < 0.01); at the same time, there was no publication bias in the funnel analysis literature, suggesting that the glucocorticoid group has a significant effect on IgA nephropathy with proteinuria greater than 1.50 g/d (see Table 3).

### 3.4. Efficacy Evaluation of Different Courses of Hormone Therapy

According to the analysis of the course of hormone treatment, 2 literature were included in the short course of treatment (duration <1 year) and 6 literature were included in the long course of treatment (duration ≥1 year). There was no publication bias in the funnel chart analysis. The heterogeneity test of literature data indicates that they are homogeneous. The analysis of fixed-effects model shows that the curative effect of short course and long course of hormone in the treatment of IgA nephropathy is statistically significant compared with the control group (*P* < 0.01, see Tables 4 and 5).

RETRACTED

### 3.5. Analysis of Therapeutic Effect of IgA Nephropathy Hormone with Different Blood Creatinine Levels

The level of serum creatinine in 6 literature was less than 1.50 mg/dl. The heterogeneity test was carried out. When *P* = 0.36 and *I*^*2*^ = 9.6, literature were homogeneous. Therefore, the fixed-effects model was selected for analysis. At the same time, funnel plot analysis showed that there was no publication bias in the literature. The results of meta-analysis showed that the SMD value and 95% *CI* were located on the left side of the vertical line: SMD = −0.61, 95% *CI* [−0.83, −0.38], and the difference was statistically significant (*P* < 0.01), suggesting that the glucocorticoid group had a better effect on proteinuria in IgA nephropathy patients with serum creatinine level less than 1.50 mg/dl (see Table 6). For IgA nephropathy patients with serum creatinine level greater than 1.50 mg/dl, meta-analysis is not possible because only one literature can be consulted. LV and other results show that the curative effect on proteinuria is also obvious.

### 3.6. Evaluation of the Efficacy of Hormone Combined with ACEI in the Treatment of Proteinuria

Among the 9 articles, 6 articles were treated with ACEI. Funnel plot analysis showed no publication bias. Six literature were tested for heterogeneity: *P* = 0.25 > 0.10 and *I*^*2*^ = 25%. There was homogeneity, which was analyzed by fixed-effects model. The results showed that the SMD value and 95% *CI* were on the left side of the vertical line: SMD = −0.52, 95% *CI* [−0.72, −0.32], and the difference was statistically significant (*P* < 0.01), suggesting that the efficacy of hormone combined with ACEI in the treatment of IgA nephropathy was better than that of the control group with ACEI alone (see Table 7).

## 4. Discussion

Glucocorticoids have anti-inflammatory, antiallergic, and immunosuppressive effects. They are widely used in the treatment of immune-mediated inflammatory reactions, including kidney diseases. Many previous studies have shown that glucocorticoids can effectively reduce urinary protein excretion and slow down the progress of kidney disease [21]. Therefore, during diagnosis and follow-up, proteinuria, blood pressure, EGFR, hematuria, and other indicators were observed to evaluate the risk of progression of nephropathy and judge the prognostic effect of glucocorticoid treatment [5, 11]. Proteinuria is an important factor determining the prognosis of IgA nephropathy. Therefore, we used proteinuria index for comprehensive analysis to evaluate the efficacy of glucocorticoid in the treatment of IgA nephropathy [22]. From the analysis of the overall efficacy evaluation of proteinuria, except that there are two literature that believe that glucocorticoids have no significant difference in improving the therapeutic effect of proteinuria compared with the control group, the others believe that the efficacy is better than the control group. The overall evaluation shows that glucocorticoids have a definite effect on proteinuria. Considering the different results of the two literature, the specific original data of patients' proteinuria levels are not provided in the literature, so the reason could not be further analyzed.

RETRACTED

Our analysis shows that glucocorticoid has obvious therapeutic effect on various degrees of proteinuria at the boundary of 1.50 g/d proteinuria, so we cannot deny the efficacy of glucocorticoid in IgA nephropathy patients with mild-to-moderate proteinuria [4]. The literature does not describe the side effects of glucocorticoid treatment. Without considering the side effects, glucocorticoid treatment can be applied to IgAN with mild-to-moderate proteinuria, but there is still a lack of large sample correlation test. From the perspective of the decrease level of urinary protein, it can be seen that, in the literature analysis of urinary protein greater than 1.50 g/d, the maximum decrease of urinary protein in microalbumin test is 1.43 g/d [23].

In Moriyama T.'s work, it is 1.87 g/d: in the literature analysis of urinary protein volume less than 1.50 g/d, the maximum decrease of urinary protein volume in Shoji T.'s test is 0.50 g/d, and in Koike M.'s work it is 0.98 g/d: intuitively compared with the value of reducing urinary protein volume, it seems that the greater the urinary protein volume, the better the hormone treatment effect [24, 25]. However, due to different sample sizes, the hormone dosage and course of treatment are not uniform; the original data of urinary protein quantity are not provided, so they can only be roughly calculated. In the future, large-sample targeted tests need to be carried out. The patients with IgA nephropathy with blood creatinine less than or greater than 1.50 mg/dl were grouped and evaluated. Only one literature in the group with blood creatinine greater than 1.50 mg/dl met the inclusion criteria. The conclusion was that the effect of hormone treatment was better than that in the nonhormone group [25]. Six literature were included in the group with blood creatinine less than 1.50 mg/dl, and the effects were obvious [10]. When both are effective for proteinuria, it is difficult to determine which group of patients is more suitable for hormone treatment, because the sample sizes of the two groups are very different, and the original data of proteinuria are not provided, so it is impossible to compare the differences between the two groups.

RETRACTED

Taking drug application as an intervention factor for subgroup analysis, we will elaborate the course of drug application and the efficacy of combined ACEI on proteinuria [7]. Among them, two literature were included in the application of hormone short course of treatment (<1 year) [10]. It was concluded that the therapeutic effect of hormone group on protein urine was better than that of nonhormone group. Due to the relatively insufficient sample sizes of the two literature, the short-term effect was considerable, and the long-term effect should be further understood. In the case of long-term application of hormone (≥1 year), the effect of hormone treatment is also obvious, but the side effects brought by long-term application of hormone are not considered, so it is impossible to weigh the effect of long-term application [2]. For long-term application and short-term application, it is difficult to determine which effect is better, because the original data of proteinuria are not provided, and the sample size is not equal or relatively insufficient, so it is impossible to compare the efficacy differences. Without considering the toxicity, some literature show that long-term application of glucocorticoids can delay the progression to end-stage renal failure. In the analysis results of intensive support therapy (combined application of hormone and ACEI), it is considered that intensive support therapy has an advantage in the treatment of IgA nephropathy in proteinuria. In this analysis, the combined application of hormone and ACEI has effectively reduced the level of proteinuria, because there is an international consensus on the role of ACEI in reducing urinary protein; therefore, whether the decrease of proteinuria level is caused by hormone treatment or the combined effect of hormone and ACEI needs to be further proved by multicenter and large-sample clinical randomized controlled trials [10]. IgA nephropathy is a progressive disease, and there are many factors affecting its prognosis. Clinically, we should comprehensively consider many factors such as the patient's clinical manifestations, pathological changes, laboratory examination results, timely and reasonable diagnosis and treatment, genetics and environment, and the patient's self-care, actively carry out clinical and basic research and take effective intervention and treatment measures, and delay or reverse the progression of IgA nephropathy.

After treatment or during follow-up, the level of proteinuria and the risk of entering ESRD in the treated group were significantly lower than those in the control group. Glucocorticoid therapy can reduce swelling and diuresis, eliminate proteinuria, and improve prognosis. In the treatment of IgA nephropathy with glucocorticoid, some authors believe that patients with IgA disease at risk of progressive renal failure (such as massive proteinuria) should be actively treated. This systematic retrospective study, including nine randomized controlled trials of more than 500 patients, provides evidence that a relatively short course of glucocorticoid therapy for IgA nephropathy reduces the risk of renal failure by two-thirds compared with supportive therapy or angiotensin-converting enzyme inhibitor therapy alone [10, 26]. Consistent with this conclusion, glucocorticoid treatment also reduced proteinuria in patients with IgA nephropathy (95% *CI*, −0.63 ∼ −0.29 g/d). These results were mainly provided by two studies, one of which did not include the best antiproteinuria and antihypertensive treatment [6]. In addition, patients with adverse events of glucocorticoid therapy, including diabetes, weight gain, and Cushing syndrome, are at increased risk in most of the trials, while the risk of other patients with more serious adverse events remains unclear. This meta-analysis has several important advantages, such as using a rigorous method, including more studies than previous reviews, focusing on clinical key results and renal failure, and tabulating adverse events. This analysis studies the potential value of glucocorticoid as a short-term treatment scheme (about 6 months). This treatment scheme is cheap and well tolerated. It has great prospects as a treatment that can greatly reduce the burden of ESRD worldwide. Due to the lack of research quality and follow-up time, this systematic evaluation cannot replace the need for large-scale clinical trials. It is still too early to use glucocorticoids as a routine treatment guide for IgA nephropathy for many reasons. At present, the available data research is small sample and short-term. It is usually carried out in a single center. The quality of the research is not optimal, and there is no continuous collection of data on side effects. Whether increasing immunosuppressive therapy can increase the benefit of patients after supporting treatment optimization remains unclear. Therefore, the balance of benefits and risks is still unclear, and the indications for hormone treatment of IgA nephropathy are still unclear.

RETRACTED

The deficiency of this meta-analysis is that some literature information is incomplete: (1) the level of proteinuria before treatment is not clearly marked. For example, Uzu T., Moriyama T., Lv J. C., and Manno C. do not describe the initial amount of proteinuria, and only the indicators of proteinuria after treatment are given. (2) There are few prognostic indicators or incomplete data, such as serum creatinine and creatinine clearance, or the initial data are not provided. (3) The original data of basic blood pressure were not described in the literature, especially for the combined application of hormone and ACEI. (4) The duration of follow-up and the number of lost visits were not clearly counted. For example, Uzu T., Moriyama T., Lv J. C., and Manno C. did not describe the number of lost visits. (5) The basic condition data of the control group are incomplete; for example, the drug dose, name, and course of treatment of the control group are not clear. (6) There is no information on hormone side effects, such as progressive hematuria and obesity [23]. (7) The sample size is relatively small, for example, 8 patients in Shoji T.'s control group and 11 patients in observation group. (8) There is no mention of influencing factors, such as blood pressure, gender, age, and race, which affects the reliability of the conclusion. Therefore, we still need to further conduct multicenter and large-sample clinical randomized controlled trial research and long-term follow-up and obtain accurate and effective information for clinical guidance in the future.

## 5. Conclusion

The overall efficacy of glucocorticoid in the treatment of IgA nephropathy is accurate. Hormone treatment is effective for different degrees of IgA nephropathy. Considering that there is no significant effect on the efficacy of different courses of treatment, it is suggested that the course of hormone treatment be appropriately shortened. Hormone combined with ACEI can reduce proteinuria more effectively than ACEI drugs alone.

## Figures and Tables

**Table 1:** Overall efficacy of hormone in the treatment of IgA nephropathy proteinuria.

Glucocorticoid group				Control group			Std. mean difference	
Study or subgroup	Mean	SD	Total	Mean	SD	Total	Weight	IV, fixed, 95% *CI*
Kobayashi et al., 1996	0.8	0.5	20	1.5	1.3	26	8.6%	−0.67 [−1.27,−0.07]
Shoji et al., 2000	0.29	0.23	11	0.71	0.39	8	2.9%	−1.31 [−2.33,−0.29]
Locatelli et al., 2001	0.67	0.5	43	1.48	1.87	43	16.5%	−0.59 [−1.02,−0.15]
Uzu et al., 2003	−1.26	0.56	23	−0.86	0.45	22	8.4%	−0.77 [−1.38,−0.16]
Moriyama et al., 2004	1.02	0.98	20	1.28	2.19	40	10.7%	−0.14 [−0.67, 0.40]
Hogg et al., 2006	−1.26	0.56	34	−0.86	0.45	31	12.1%	−0.77 [−1.28, −0.27]
Koike et al., 2008	0.31	0.51	24	0.68	0.69	24	9.2%	−0.60 [−1.18, −0.02]
Lv et al. 2009	−2.5	0.9	33	−2	0.8	30	12.1%	−0.58 [−1.08, −0.07]
Manno et al., 2009	1.2	2.5	48	1.4	2.3	49	19.5%	−0.08 [−0.48, 0.32]
Total (95% CI)			256			273	100.0%	−0.51 [−0.68, −0.33]

Heterogeneity: Chi-squared = 10.93, df = 8 (*P* = 0.21); *F* = 27%; test for overall effect: *Z* = 5.65 (*P*＜0.00001).

RETRACTED

**Table 2:** Effect of glucocorticoid on IgA nephropathy patients with proteinuria less than 1.50 g/d.

Glucocorticoid group				Control group			Std. mean difference	
Study or subgroup	Mean	SD	Total	Mean	SD	Total	Weight	IV, fixed, 95% *CI*
Shoji et al., 2000	0.29	0.23	11	0.71	0.39	8	24.3%	−1.31 [−2.33,−0.29]
Koike et al., 2008	0.31	0.51	24	0.68	0.69	24	75.7%	−0.60 [−1.18,−0.02]
Total (95% CI)			35			32	100.0%	−0.77 [−1.28,−0.27]

Heterogeneity: Chi' = 1.40, df = 1 (*P* = 0.24); *I*^*2*^ = 29%; test for overall effect: *Z* = 3.00 (*P* = 0.003).

**Table 3:** Effect of glucocorticoid on IgA nephropathy patients with proteinuria greater than 1.50 g/d.

Glucocorticoid group				Control group			Std. mean difference	
Study or subgroup	Mean	SD	Total	Mean	SD	Total	Weight	IV, fixed, 95% *CI*
Locatelli et al., 2001	0.67	0.5	43	1.48	1.87	43	60.7%	−0.59 [−1.02,−0.15]
Moriyama et al., 2004	1.02	0.98	20	1.28	2.19	40	39.3%	−0.14 [−0.67, 0.40]
Total (95% CI)			63			83	100.0%	−0.41 [−0.75,−0.07]

Heterogeneity: Chi' = 1.64, df = 1 (*P* = 0.20); *I*^*2*^ = 39%. Test for overall effect: *Z* = 2.38 (*P* = 0.02).

**Table 4:** Effect of short-term (<1 year) course of glucocorticoid on proteinuria in IgA nephropathy.

Glucocorticoid group				Control group			Std. mean difference	
Study or subgroup	Mean	SD	Total	Mean	SD	Total	Weight	IV, fixed, 95% *CI*
Locatelli et al., 2001	0.67	0.5	43	1.48	1.87	43	66.4%	−0.59 [−1.02,−0.15]
Uzu T et al., 2003	−1.26	0.56	23	−0.86	0.45	22	33.6%	−0.77 [−1.38,−0.16]
Total (95% CI)			66			65	100.0%	−0.65 [−1.00,−0.30]

Heterogeneity: Chi' = 0.24, df = 1 (*P* = 0.63); *I*^*2*^ = 0%. Test for overall effect: *Z* = 3.61 (*P* = 0.0003).

**Table 5:** Effect of long-term (≥1 year) course of glucocorticoid on proteinuria in IgA nephropathy.

Glucocorticoid group				Control group			Std. mean difference	
Study or subgroup	Mean	SD	Total	Mean	SD	Total	Weight	IV, fixed, 95% *CI*
Kobayashi et al., 1996	0.8	0.5	20	1.5	1.3	26	15.4%	−0.67 [−1.27,−0.07]
Shoji et al., 2000	0.29	0.23	11	0.71	0.39	8	5.3%	−1.31 [−2.33,−0.29]
Moriyama et al., 2004	1.02	0.98	20	1.28	2.19	40	19.2%	−0.14 [−0.67, 0.40]
Hogg et al., 2006	−1.26	0.56	34	−0.86	0.45	31	21.7%	−0.77 [−1.28, −0.27]
Koike et al., 2008	0.31	0.51	24	0.68	0.69	24	16.5%	−0.60 [−1.18, −0.02]
Lv et al., 2009	−2.5	0.9	33	−2	0.8	30	21.8%	−0.58 [−1.08, −0.07]
Total (95% CI)			142			159	100.0%	−0.59 [−0.83, −0.36]

Heterogeneity: Chi' = 5.21, df = 5 (*P* = 0.39); *F* = 4%. Test for overall effect: *Z* = 4.92 (*P*＜0.00001).

**Table 6:** Effect of glucocorticoid on IgA nephropathy proteinuria with blood creatinine level less than 1.50 mg/dl.

Glucocorticoid group				Control group			Std. mean difference	
Study or subgroup	Mean	SD	Total	Mean	SD	Total	Weight	IV, fixed, 95% *CI*
Shoji et al., 2000	0.29	0.23	11	0.71	0.39	8	4.9%	−1.31 [−2.33,−0.29]
Locatelli et al., 2001	0.67	0.5	43	1.48	1.87	43	27.7%	−0.59 [−1.02,−0.15]
Uzu et al., 2003	−1.26	0.56	23	−0.86	0.45	22	14.0%	−0.77 [−1.38,−0.16]
Moriyama et al., 2004	1.02	0.98	20	1.28	2.19	40	17.9%	−0.14 [−0.67, 0.40]
Hogg et al., 2006	−1.26	0.56	34	−0.86	0.45	31	20.2%	−0.77 [−1.28, −0.27]
Koike et al., 2008	0.31	0.51	24	0.68	0.69	24	15.4%	−0.60 [−1.18, −0.02]
Total (95% CI)			155			168	100.0%	−0.61 [−0.83, −0.38]

Heterogeneity: Chi' = 5.47, df = 5 (*P* = 0.36); *F* = 9%. Test for overall effect: *Z* = 5.24 (*P*＜0.00001).

RETRACTED

**Table 7:** Effect of hormone combined with ACEI drugs on proteinuria in patients with IgA nephropathy.

Glucocorticoid group				Control group			Std. mean difference	
Study or subgroup	Mean	Sd	Total	Mean	Sd	Total	Weight	IV, fixed, 95% *CI*
Kobayashi et al., 1996	0.8	0.5	20	1.5	1.3	26	11.1%	−0.67 [−1.27, −0.07]
Locatelli et al., 2001	0.67	0.5	43	1.48	1.87	43	21.4%	−0.59 [−1.02,−0.15]
Uzu et al., 2003	−1.26	0.56	23	−0.86	0.45	22	10.8%	−0.77 [−1.38, −0.16]
Moriyama et al., 2004	−1.26	0.56	34	−0.86	0.45	31	15.7%	−0.77 [−1.28, −0.27]
Lv et al., 2009	−2.5	0.9	33	−2	0.8	30	15.7%	−0.58 [−1.08,−0.07]
Manno et al., 2009	1.2	2.5	48	1.4	2.3	49	25.3%	−0.08 [−0.48, 0.32]
Total (95% CI)			201			201	100.0%	−0.52 [−0.72, −0.32]

Heterogeneity: Chi' = 6.63, df = 5 (*P* = 0.25); *F* = 25%. Test for overall effect: *Z* = 5.06 (*P*＜0.00001).

## Data Availability

The data used to support this study are available from the corresponding author upon request.
